The article "Inter-Relationship Between a Transcriptional Regulator of Flagella Genes cj0440c and Thiamine Metabolic Pathway in Campylobacter jejuni" was retracted in 2024. Reasons: signs of a paper mill; suspected computer-generated content; unreliable results or conclusions; concerns about the data.

# Inter-Relationship Between a Transcriptional Regulator of Flagella Genes *cj0440c* and Thiamine Metabolic Pathway in *Campylobacter jejuni*

**DOI:** 10.1155/2022/4539367

**Published:** 2022-08-21

**Authors:** Muhammad Abu Bakr Shabbir, Aziz Ul-Rahman, Abdur Rauf Khalid, Nabeel Ijaz, Muhammmad Tahir Aleem, Saeed Ahmed, Abdulaziz Alouffi, Waqas Ahmed, Faiza Aslam, Muhammad Kashif Maan, Adnan Hassan Tahir, Muhammad Waqar Aziz, Mashal M. Almutairi, Haihong Hao

**Affiliations:** ^1^Institute of Microbiology, University of Veterinary and Animal Sciences Lahore, 54600, Pakistan; ^2^Department of Pathobiology, Faculty of Veterinary and Animal Sciences, MNS University of Agriculture, Multan 66000, Pakistan; ^3^Department of Livestock and Poultry Production, Faculty of Veterinary Sciences, Bahauddin Zakariya University, Multan, Pakistan; ^4^Department of Clinical Sciences, Faculty of Veterinary Sciences, Bahauddin Zakariya University, Multan, Pakistan; ^5^MOE Joint International Research Laboratory of Animal Health and Food Safety, College of Veterinary Medicine, Nanjing Agricultural University, Nanjing 210095, China; ^6^Department of Biological Sciences, National University of Medical Sciences (NUMS), Islamabad, Pakistan; ^7^King Abdulaziz City for Science and Technology, Riyadh 12354, Saudi Arabia; ^8^Department of Biomedical and Diagnostic Science, University of Tennessee Knoxville, USA; ^9^Livestock and Dairy Development Department, Lahore 54000, Pakistan; ^10^Department of Veterinary Surgery and Pet Sciences, Faculty of Veterinary Science, University of Veterinary and Animal Sciences, Lahore, Pakistan; ^11^Department of Clinical Sciences, Faculty of Veterinary and Animal Sciences, PMAS-Arid Agriculture University Rawalpindi, Pakistan; ^12^Department of Pharmacology and Toxicology, College of Pharmacy, King Saud University, Riyadh 11451, Saudi Arabia; ^13^MOA Laboratory for Risk Assessment of Quality & Safety of Livestock & Poultry Products, Huazhong Agricultural University, Wuhan 430070, China

## Abstract

*Campylobacter jejuni* is a major cause of gastroenteritis in humans. It has been reported that the pathogenesis of *C. jejuni* is closely related to the formation, adhesion, and invasion of flagella toxin in host epithelial cells. A putative transcriptional regulator, known as *cj0440c*, is thought to be involved in the regulation of flagellar synthesis. However, confirmation of this hypothesis requires deep insight into the regulation mechanism of *cj0440c* and its possible relationship with different antibiotics. Therefore, the study explained here was designed to determine the relationship and function (phenotypically and genotypically) of *cj0440c* in the flagellar synthesis of *C. jejuni* NCTC11168. The study determined the mode of expression of *cj0440c* and flagella-related genes under exposure to various drugs. To verify the involvement of *cj0440c* protein in the metabolic pathway of thiamine, an enzymatic hydrolysis experiment was performed and analyzed through the application of mass spectrometry. The overexpression vector of *C. jejuni* NCTC11168 was also constructed to find out whether or not target genes were regulated by *cj0440c*. The findings of the study showed that *cj0440c* and other flagella-related genes were expressed differentially under the influence of various antibiotics including erythromycin, tylosin, azithromycin, gentamicin, etimicin, enrofloxacin, gatifloxacin, tetracycline, and tigecycline. The analysis showed that the *cj0440c* protein did not catalyze the degradation of thiamine. In conclusion, the study aids in the understanding of the inter-relationship between the regulatory mechanism of flagella genes and the thiamine metabolic pathway.

## 1. Introduction

*Campylobacter jejuni* (*C. jejuni*) is a pathogenic bacterium that is considered a major cause of food-borne diarrhea around the globe [1]. It is estimated that more than 400 million people each year are exposed to these bacteria and, as a consequence, develop gastroenteritis [2]. Humans may be infected via the consumption of contaminated poultry meat, milk, or water [3, 4]. Outbreaks of *C. jejuni* infection in humans are relatively rare. However, *Campylobacter* infection has serious consequences in those with autoimmune-mediated diseases such as Guillain-Barre syndrome and Miller-Fisher syndrome [5]. It has been found that the pathogenesis of *Campylobacter* is closely related to the formation, adhesion, and invasion of the toxin of the flagella in the host epithelial cells [6]. The motility of the flagella helps the bacteria to cross the membrane of intestinal epithelial cells [7]. Therefore, the role of flagella in *C. jejuni* virulence should not be underestimated.

The synthesis of *C. jejuni* flagella is a complex process; more than 50 genes such as *flgS (Cj0793)*, *flgR (CJ1024)*, and *fliA (Cj0061)* are involved in their synthesis and regulation [8]. Three sigma factors (*σ^70^*, *σ^54^*, and *σ^28^*) are involved in the regulation of flagellar synthesis in *C. jejuni*. However, research on the regulatory mechanism of flagella has focused on the deletion mutation of known genes, and information is scarce regarding the *cj0440c* gene. Bioinformatic analysis reveals that *cj0440c* is a putative transcriptional regulator that encodes a TEN/THI-4 protein family, but the molecular function of this family has not been determined. This gene (*cj0440c*) is present upstream of *cj0441* (which creates an acyl carrier protein, acpP) [9] and downstream of the *cj0437*-*cj0439* operon, which plays a pivotal role in the susceptibility of *Campylobacter* to hydrogen peroxide (H_2_O_2_) [10, 11]. Hence, genes that lie both upstream and downstream of *cj0440c* are essential for *Campylobacter*'s survival, growth, colonization, and pathogenesis. Although the *cj0440c* gene is present at opposite ends of the DNA coding strand, it can be divergently transcribed with its up-and-downstream genes and probably acts as a transcriptional regulator for several genes that are involved in the biosynthesis of flagella. However, the biological functions of *cj0440c* in *C. jejuni* are mostly unknown.

Due to the involvement of the *cj0440c* gene in the regulation of flagellar synthesis and the lack of information on the possible influence of antibiotic resistance, the study explained here was designed to determine the relationship and function (phenotypically and genotypically) of *cj0440c* in the flagellar synthesis of *C. jejuni* NCTC11168. To achieve that, the expression of *cj0440c* and other flagella genes during exposure to eight different kinds of antibiotics was detected through the use of reverse-transcription polymerase chain reaction (RT-PCR) preliminarily to detect the relationship between *cj0440c* and flagella genes. The *cj0440c* protein was expressed and purified, and a digestion experiment was designed that employed thiamine as the substrate to determine whether or not *cj0440c* was a thiaminase and can regulate directly the expression of flagella genes.

## 2. Materials and Methods

### 2.1. Bacterial Strains, Plasmids, and Culture Conditions

The *C. jejuni* NCTC11168 strain that was designated as sensitive (S) was obtained from the Chinese Centre for Disease Control and Prevention. The *Escherichia coli* strains and plasmids that were used in this study and their sources are listed in Table 1. *Campylobacter* strains were grown on plates that contained Skirrow *Campylobacter* selective agar (Hopebio, Qingdao, China) and were supplemented with 5% sterile defibrinated sheep blood at 42 °C under a microaerobic environment (85% N_2_, 10% CO_2_, and 5% O_2_). The *C. jejuni* NCTC11168 strain that was designated as resistant (R), which was resistant to different kinds of antibiotics, was procured from our laboratory (the China Ministry of Agriculture Laboratory for Risk Assessment of Quality and Safety of Livestock and Poultry Products, Huazhong Agricultural University, Wuhan, China). *E. coli* cells were grown at 37 °C in a shaking incubator (200 rpm) in Luria-Bertani (LB) medium. When necessary, LB media were supplemented with kanamycin (30 *μ*g/ml) or ampicillin (100 *μ*g/ml).

### 2.2. Antimicrobial Susceptibility Assessment

The minimal inhibitory concentrations (MICs) of S and R against nine commercially available and frequently practiced antimicrobials, which were erythromycin (Ery), tylosin (Tyl), azithromycin (Azi), gentamicin (Gen), etimicin (Eti), enrofloxacin (Enr), gatifloxacin (Gati), tetracycline (Tet), and tigecycline (Tige), were determined by use of the broth microdilution susceptibility method, as described previously by the Clinical and Laboratory Standards Institute [12]. *C. jejuni* ATCC33560 was used as the quality control strain. The experiment was performed in triplicate.

The mutant prevention concentration (MPC) was defined as the lowest concentration of drug that prevented bacterial colony formation in a culture that contained >10^10^ bacteria. The determination was similar to that for the MIC, except that >10^10^ cells were tested at high drug concentrations (from 1 MIC to 128 MIC) and agar plates were used. Inoculated plates were incubated for 72 h. The minimum drug concentration that led to nonbacterial growth was the provisional MPC (MPC_pr_). The mutant selection window (MSW) was the drug concentration range between the MIC and the MPC.

### 2.3. Detection of Expression of Flagella Genes in *C. jejuni* by RT-PCR

Both strains (S and R) were induced by the addition of 0.5MPC of each of the eight antibiotics. The total RNA from each sample was extracted using the RNAprep pure cell/bacteria kit (Tiangen Biotech, Beijing, China). The quality and quantity of the RNA were determined by the application of formaldehyde denaturing gel electrophoresis and the use of a Nanodrop TM 2000 Spectrophotometer (Thermo Fisher Scientific, Waltham, MA, USA). The cDNA was synthesized from the extracted RNA using a HiScript II one-step RT-PCR kit (Nanjing Vazyme Biotech Co, Nanjing, China).

The batches of cDNA of nine antibiotic-resistant bacteria and standard bacteria were subjected to RT-PCR to determine the expression of the flagellar genes, according to a previously described study [13]. Briefly, the PCR amplification was performed in the IQ5 Multicolor Real-time PCR Detection System (Bio-Rad Laboratories, Hercules, CA, USA). The cycling conditions were as follows: 3 min of pre-incubation at 95 °C, followed by 45 cycles of 10s at 95 °C and 40s at 52 °C. The primer sets used for specific genes (*cj0440c*, *cj1339c*, *cj1338c, cj0043*, *cj0697*, and *16S*) are listed in Table 2. It was decided to use 16S rDNA as an internal control for normalization. The experiment was performed in triplicate to obtain an average value for the fold change. A *t*-test was performed to analyze the significant difference between resistant bacteria and standard bacteria.

### 2.4. Construction of *cj0440c* Overexpression Mutants in *C. jejuni* NCTC11168

The DNA fragment of the *cj0440c* gene and promoter *CmeABC* was amplified from the *C. jejuni* NCTC11168 genome using Taq polymerase (Takara, Kusatsu, Shiga, Japan) with primers of *cj0440c*-F/R and C*meABC*-F/R (Table 2). The *cj0440c*-F/R carried endonuclease restriction sites of *Sac* I and *Sac* II, while *CmeABC*-F/R carried endonuclease restriction sites of Sac I and *Spe* I. PCRs were performed in a total volume of 20 *μ*l using 0.5 *μ*l of each primer (10 *μ*M), 2 *μ*l of Taq polymerase buffer (10×), 1.6 *μ*l of deoxynucleoside triphosphates (2.5 mM), 0.2 *μ*l of Taq polymerase, and 200 ng of DNA template. The amplification program was as follows: initial denaturation at 95 °C for 5 min, denaturation at 95 °C for 30s, and annealing at 52 °C for 30s, followed by 35 cycles of extension at 72 °C for 1 min and an additional final extension at 72 °C for 5 min. PCR products were evaluated on a 1% agarose gel under ultraviolet light in the presence of ethidium bromide. After the reaction, the PCR products were analyzed on agarose gel, and the desired gene fragments were excised and purified through the use of a gel extraction kit (Omega Bio-tek Inc. Georgia, USA).

T4 DNA ligase enzyme (Takara, Kusatsu, Shiga, Japan) was used to connect *cj0440c* and *CmeABC* fragments by the same restriction sites (*Sac* I) to gain a new fragment *Cme440.* This new fragment was then cloned into a pMD19-T sample vector (Takara, Kusatsu, Shiga, Japan) to generate plasmid *T-Cme440*. Enzymatic double digestion (which involves cutting DNA with two restriction enzymes simultaneously) was used for Spe I and Sac II. A similar action was replicated on the vector pRY112. Insertion was performed at 16 °C using the T4 DNA ligase enzyme. The ligation product was transformed into DH5*α* by heat shock (at 4 °C for 30 min, 42 °C for 90s, and 4 °C for 2 min). Afterward, the transformed cells were restored through the addition of LB liquid medium to the transformants, and the mixture was incubated for 2 h. Bacteria were collected through the use of low-speed centrifugation. Finally, bacterial pellets were added to an LB medium that contained chloramphenicol to produce the recombinant clones that contained the vector. The clones were sent to the company for sequencing and the right plasmid was named *pRY-Cme440*.

### 2.5. Cloning, Expression, and Purification of *cj0440c* in *E. coli*

The size of the target gene *cj0440c* (Gene ID: 904765) was 666 bp. The DNA fragment of the *cj0440c* gene was amplified from the *C. jejuni* NCTC11168 genome through the use of Taq polymerase (Takara, Kusatsu, Shiga, Japan) with primers of *cj0440c*-F1/R1 (Table 2) that carried endonuclease restriction sites of BamH I and Xho I. The vector (*pET28a*) was of size 5369 bp and carried a kanamycin resistance gene and different restriction sites for various enzymes. The expression vector was constructed through the use of the method described above and was named the expression vector *P-440*.

### 2.6. Inducible Expression and Purification of *cj0440c* Protein

The expression host *E. coli* BL21 was used for the expression of recombinant protein *cj0440c*. Induction of the bacteria that contained *P-440* was performed by overnight culture in the presence of 50 *μ*g/ml kanamycin. Bacterial culture (200 *μ*l) was grown in broth media and transferred to 20 ml of fresh liquid medium. The growth of bacterial culture was monitored by an optical density (OD) spectrophotometer at 600 nm. Isopropyl-*β*-d-thiogalactoside (IPTG) was added when the OD_600_ value reached 0.6 to induce the protein expression. The best conditions for expression of cj0440c protein were found to be 0.1 mM IPTG at 25 °C for 20 h with the use of *E. coli* BL21 (DE3) cells.

The recombinant protein contained N-terminal 6 × His tags and C-terminal 6 × His tags. It was purified from the cell lysate through the use of nickel-nitriloacetic acid (Ni-NTA) affinity chromatography. The *E. coli* BL21 cells, which contained *P-440* after induction, were harvested by centrifugation at 4000 rpm for 20 min. The cells were resuspended in ice-cold phosphate-buffered saline (PBS) and sonicated at 50% power for 30 min. The cell lysates were centrifuged at 12000 rpm for 30 min at 4 °C. The supernatant was incubated with 100 *μ*l Ni-NTA Sepharose (GE Healthcare, Chicago, Il, USA) in 1.5 ml tubes at 4 °C for 2 h in a shaking incubator. The supernatant was washed with 1 ml of Ni-NTA wash buffer (50 mM NaH_2_PO_4_, pH 8.0, 300 mM NaCl, and 300 mM imidazole). Next, the bound proteins were eluted in 1 ml of Ni-NTA elution buffer (50 mM NaH_2_PO_4_, pH 8.0, 300 mM NaCl, and 500 mM imidazole). The eluted protein was run through a 12% sodium dodecyl sulfate-polyacrylamide gel electrophoresis (SDS-PAGE) system and then transferred to a polyvinylidene difluoride (PVDF) membrane and immunoblotted with anti-His antibody.

### 2.7. Detection of the Role of *cj0440c* in Thiamine Metabolism

TenA can catalyze thiamine degradation to 4-methyl-5-(2-hydroxyethyl) thiazole (THZ) and 4-amino-5-hydroxymethyl-2-methylpyrimidine (HMP) (Figure 1).

For qualitative assessment, thiaminase activity of *cj0440c* was identified by incubating different concentrations (15 *μ*M, 20 *μ*M, 25 *μ*M, or 30 *μ*M) of *cj0440c* and thiamine (2.5 mM) at room temperature in 50 mM *tris*(hydroxymethyl)aminomethane (tris buffer) (pH 8.0). A 100 *μ*l aliquot of this reaction mixture was removed after 5 h and quenched by heating at 95 °C for 2 min. The reaction was repeated without cj0440c to produce the control, and then the compounds were analyzed by mass spectrometry (MS).

## 3. Results

### 3.1. Antimicrobial Susceptibility of *C. jejuni* NCTC11168 (S and R Strains)

The susceptibility of *C. jejuni* NCTC11168 (S and R strains) to each of nine antibiotics was determined. As expected, the *C. jejuni* NCTC11168 (R) showed higher resistance to the nine tested antibiotics than the S strain, as shown in Table 3. Likewise, high MPC and MSW were observed in the *C. jejuni* NCTC11168 (R) strain when compared with the S strain.

### 3.2. Expression of *cj0440c* and Other Flagella-Related Genes in *C. jejuni* NCTC11168 (S and R Strains) Exposed to Antibiotics

The expression of flagella-related genes was measured through the use of real-time quantitative RT-PCR (qRT-PCR) during exposure to the macrolide, aminoglycoside, quinolone, and tetracycline groups of antibiotics. Among these genes, *16S* rDNA was used as an internal control, *cj1338c* and *cj1339c* were those that transcribed the filament proteins, *cj0043* was the gene for the flagellar hook protein, and *cj0697* was the gene for the flagellar basal body protein. It is of note that these four genes are distributed in every part of the flagella. A trend toward increased expression of all genes including *cj0440c* in the presence of macrolides (Ery and Azi), aminoglycosides (Gen and Eti), quinolones (Enr and Gati), and tetracyclines (Tet and Tige) was observed in the study (Figures 2(a)–2(d)).

### 3.3. The Western Blot Analysis of *cj0440c* Protein

A western blot analysis revealed the increased expression of protein under the influence of IPTG (Figure 3). The best conditions for induction of *cj0440c* protein were 20 h in 0.1 mM IPTG at 25 °C; the best purification conditions for this protein were its elution in 500 mM imidazole.

### 3.4. Reaction of *cj0440c* with Thiamine

MS was used to determine the products of the reaction of catalyzed thiamine with different concentrations of *cj0440c* protein (Figures 4(a)–4(e)).  Figure 4(a) represents the blank group that is without *cj0440c*. The molecular weight of thiamine is 337 kDa, that of THZ is 143 kDa and that of HMP is 139 kDa. There was no difference between the results for the experimental group and those for the blank group. MS analysis showed that the *cj0440c* protein did not catalyze the degradation of thiamine.

## 4. Discussion

Over the last decade, *C. jejuni* has become considered one of the leading causes of food poisoning in many countries including those in Europe [14]. Because of its public health significance, it is important to study the pathogenic mechanisms that are adopted by this bacterium. Among pathogenic mechanisms, the formation of flagella is key, as they aid bacterium motility, biofilm formation, adherence, and invasion into the host cell [15]. The *cj0440c* gene, a putative transcriptional regulator of several flagella-related genes, and its role in the biosynthesis of flagella is not fully understood. Therefore, the study described here was conducted to determine the association of this transcriptional regulator with other flagella-related genes. The determination was performed with the use of RT-PCR. It was observed through the use of MS analysis that *cj0440c* had no role in thiamine hydrolysis. It was also found that *cj0440c* was not involved directly in the regulation of flagella genes. Increased expression of *cj0440c* and other flagellar genes (*cj1338c*, *cj1339c*, *cj0697*, and *cj0043*) was found in *C. jejuni* NCTC11168 (S and R strains) upon exposure of the bacterium to eight different kinds of antibiotics. Flagella-related genes such as *cj1338c*, *cj1339c*, *cj0697*, and *cj0043* are distributed in every part of the flagella, including the basal body, the hook, and the filament. These genes along with a putative transcriptional regulator (*cj0440c*) were upregulated upon exposure to antibiotics.

The outcomes of this study are in agreement with previous observations on the upregulation of the *cj0440c* gene in the Ery^r^*C. jejuni* [16]. It is known that bacteria suffer a fitness cost during antibiotic resistance; however, numerous other factors are involved in the compensation for the adaptation weakness [14–18]. In this study, increased expression of flagella-related genes and *cj0440c* suggest that the putative transcriptional regulator may affect morphological changes of the flagella by taking part in the regulation of filament. One possible explanation is that *cj0440c* may be involved in compensating for the fitness cost of various antibiotics *via* a positive relationship with flagella-related genes. These findings are in agreement with those of a previous study [19].

It has been reported that the *cj0440c* gene may have a role in encoding the TenA/PQQC/THI-4 family of proteins. TenA proteins enhance the expression of extracellular enzymes such as alkaline proteases, levansucrases, and neutral proteases [20]. TenA is a thiaminase II [21], and it can catalyze the degradation of thiamine [22, 23]. This family also includes pyrroloquinoline quinone synthesis protein C (PQQC). This PQQC is a prosthetic group of numerous bacterial enzymes such as methanol dehydrogenase of methylotrophs and glucose dehydrogenase [24, 25]. Biosynthesis of PQQC in *E. coli* can be affected by the actions of the *tldD* gene, which is involved in the processing of small peptides [26]. This gene removes repression of the *cdtB* and *lgeR* genes, which may regulate some flagella genes [27]. However, the findings of the present study show that cj0440c is not an enzyme, and it cannot take part in the metabolic pathways of thiamine.

This study preliminarily explored the function of *cj0440c*; it contributed to the improvement of the genome informatics of *Campylobacter*, and it provided the theoretical basis for the study of the mechanism in *Campylobacter*. The limitation of the current study was that all the experiments were performed *in vitro*, and research methods on the regulatory mechanisms of prokaryotes are limited. Therefore, further study is required to understand the signaling pathway.

## 5. Conclusion

Owing to the potential of *Campylobacter jejuni* to cause health issues among public communities with the involvement of antibiotic resistance, the current study revealed that the transcriptional regulator known as *cj0440c* does not transcribe an enzyme; therefore, this gene may not be involved in the synthesis of thiamine. The outcome also revealed that *C. jejuni* NCTC11168 (R) showed higher resistance to the nine tested antibiotics than the S strain with increased expression of the *cj0440c* gene in the presence of macrolides, aminoglycosides, quinolones, and tetracyclines. The study aids in the understanding of the inter-relationship between the regulatory mechanism of flagella genes and the thiamine metabolic pathway.

## Figures and Tables

**Figure 1:** The degradation of thiamine into THZ and HMP catalyzing by *TenA.*

**Figure 2:** (a)–(d) The increased expression of Flagella-related genes by qRT-PCR under the exposure of different antibiotics in *C. jejuni* NCTC11168 (S & R) strains. (a) shows the increased expression of flagella-related genes under the exposure of macrolide antibiotics; (b) shows the increased expression of flagellar-related genes under the exposure of aminoglycoside antibiotics; (c) shows the increased expression of flagella-related genes under the exposure of quinolone antibiotics, and (d) shows the increased expression of flagella-related genes under the exposure of tetracycline antibiotics in *C. jejuni* NCTC11168 (S & R) strains.

**Figure 3:** The expression of protein *Cj0440c* through western blot. Lane M is protein molecular weight 116 Marker; lane 1 is *C. jejuni* NCTC1118 control before induction; lane 2 is overexpression protein after induction by IPTG, and lane 3 is a purified protein.

**Figure 4:** (a)–(e) The mass spectrogram of the product of *cj0440c* protein enzymatic hydrolysis. (a) The blank group (without *cj0440c* protein); (b) contains 15 *μ*M *cj0440c* protein; (c) contains 20 *μ*M *cj0440c* protein; (d) contains 25 *μ*M *cj0440c* protein; (e) contains 30 *μ*M *cj0440c* protein.

**Table 1:** Bacterial strain and plasmid used in the present study.

Name	Description
Bacterial strain	
NCTC 11168	*Campylobacter jejuni* NCTC 11168 (S)
NCTC 11168	*Campylobacter jejuni* NCTC 11168 (R)
ATCC 33560	*Campylobacter jejuni* ATCC 33560
DH5*α*	*E. coli* strain for DNA manipulation
BL21	*E. coli* strain for DNA manipulation
Plasmid	
pRY112	Cm-resistant *C. jejuni*/*E. coli* vector
pMD19-T simple	Amp-resistant *E. coli* vector
pET28-a	Km-resistant *E. coli* vector

**Table 2:** Primers used for qRT-PCR in the current study.

Gene	Sequence (5′-3′)
*Cj0440c*-F	CGAGCTCATGcaccaccaccaccaccacATGCTTTTCTCTAATTTAATCA
*Cj0440c*-R	TCCCCGCGGTTAAAGATTTAATTCCATTCTTAAAGAA

*CmeABC*-F	GGACTAGTTAAATGGAATCAATAGCTCCAAAGC
*CmeABC*-R	CGAGCTCCAGGGTAAGTAAAACTAAGTGGTAA

*Cj0440c*-F1	CGGGATCCATGATGCTTTTCTCTAATTTAATCA
*Cj0440c*-R1	CCCTCGAGAAGATTTAATTCCATTCTTAAAGAA

*Cj0440c*F	AGTTGCTCTTAGTGCTTGCG
*Cj0440c*R	TGCTCCCAAAAAGCCACTTC

*Cj1339c*F	TCCATTAAACGGTTGATATCTGCTT
*Cj1339c*R	AAGGCTATGGATGAGCAACTTAAAAT

*Cj0043*F	GGGTTCTCCTGTTGCAAGTGA
*Cj0043*R	GCCCCTAAAACCCCAAAAAAT

*Cj1338c*F	TTACCATTGTTGATAGCTTGACCTAAA
*Cj1338c*R	TGCTTCAGGGATGGCGATA

*Cj0697*F	TGGTTCAGACCAAAGATGGA
*Cj0697*R	TGCCAGCATTCTGAGGATTA

*16S*F	GCTCGTGTCGTGAGATGTTG
*16S*R	GCGGTATTGCGTCTCATTGTAT

**Table 3:** The MIC, MPC, and MSW results of *C. jejuni* NCTC11168 (S) and *C. jejuni* NCTC11168 (R) for nine antibiotic drugs.

Name	NCTC11168 (S)		NCTC11168 (R)			
	MIC (*μ*g/mL)	MPC	MSW	MIC (*μ*g/mL)	MPC	MSW
Erythromycin	0.125	2MIC	1-2MIC	0.5	2MIC	1-4MIC
Tylosin	0.5	2MIC	1-2MIC	2.0	4MIC	1-4MIC
Azithromycin	<0.125	2MIC	1-2MIC	0.5	4MIC	1-4MIC
Gentamicin	0.25	4MIC	1-4MIC	0.5	8MIC	1-8MIC
Etimicin	1.0	4MIC	1-4MIC	2.0	8MIC	1-8MIC
Enrofloxacin	0.125	8MIC	1-8MIC	4.0	32MIC	1-32MIC
Gatifloxacin	0.25	4MIC	1-4MIC	4.0	8MIC	1-8MIC
Tetracycline	0.125	32MIC	1-32MIC	16.0	128MIC	1-128MIC
Tigecycline	<0.125	8MIC	1-8MIC	0.25	64MIC	1-64MIC

## Data Availability

All the data are available in the manuscript.

## References

[1] Moore J. E., Corcoran D., Dooley J. S. G. (2005). Campylobacter. *Veterinary Research*.

[2] Acheson D., Allos B. M. (2001). Campylobacter jejuni infections: update on emerging issues and trends. *Clinical Infectious Diseases*.

[3] Pitkänen T. (2013). Review of Campylobacter_ spp. in drinking and environmental waters. *Journal of Microbiological Methods*.

[4] Huang H., Brooks B. W., Lowman R., Carrillo C. D. (2015). *Campylobacter* species in animal, food, and environmental sources, and relevant testing programs in Canada.

[5] Han K., Jang S. S., Choo E., Heu S., Ryu S. (2007). Prevalence, genetic diversity, and antibiotic resistance patterns of _Campylobacter jejuni_ from retail raw chickens in Korea. *International Journal of Food Microbiology*.

[6] Scanlan E., Yu L., Maskell D., Choudhary J., Grant A. (2017). A quantitative proteomic screen of the _Campylobacter jejuni_ flagellar- dependent secretome. *Journal of Proteomics*.

[7] Akahoshi D. T., Bevins C. L. (2022). Flagella at the host-microbe interface: key functions intersect with redundant responses. *Frontiers in Immunology*.

[8] Wösten M. M. S. M., Wagenaar J. A., van Putten J. P. M. (2004). The FlgS/FlgR two-component signal transduction system regulates the *fla* Regulon in *Campylobacter jejuni*. *The Journal of Biological Chemistry*.

[9] Byers D. M., Gong H. (2007). Acyl carrier protein: structure–function relationships in a conserved multifunctional protein family. *Biochemistry and Cell Biology*.

[10] Kassem I. I., Khatri M., Esseili M. A. (2012). Respiratory proteins contribute differentially to campylobacter jejuni’s survival and in vitro interaction with hosts’ intestinal cells. *BMC Microbiology*.

[11] Weingarten R. A., Taveirne M. E., Olson J. W. (2009). The dual-functioning fumarate reductase is the sole succinate: quinone reductase in Campylobacter jejuni and is required for full host colonization. *Journal of Bacteriology*.

[12] Patel J. B., Cockerill F. R., Bradford P. A. (2015). Performance standards for antimicrobial susceptibility testing: Twenty-Fifth Informational Supplement. *Clinical and Laboratory Standards Institute*.

[13] Shabbir M. A. B., Wu Q., Shabbir M. Z. (2018). The CRISPR-cas system promotes antimicrobial resistance in Campylobacter jejuni. *Future Microbiology*.

[14] Bronnec V., Turoňová H., Bouju A. (2016). Adhesion, biofilm formation, and genomic features of campylobacter jejuni Bf, an atypical strain able to grow under aerobic conditions. *Frontiers in Microbiology*.

[15] Guerry P. (2007). *Campylobacter* flagella: not just for motility. *Trends in Microbiology*.

[16] Hao H., Yuan Z., Shen Z. (2013). Mutational and transcriptomic changes involved in the development of macrolide resistance in campylobacter jejuni. *Antimicrobial Agents and Chemotherapy*.

[17] Björkman J., Andersson D. I. (2000). The cost of antibiotic resistance from a bacterial perspective. *Drug Resistance Updates*.

[18] Kugelberg E., Kofoid E., Reams A. B., Andersson D. I., Roth J. R. (2006). Multiple pathways of selected gene amplification during adaptive mutation. *Proceedings of the National Academy of Sciences*.

[19] Hao H., Fang X., Han J. (2017). Cj0440c affects flagella formation and in vivo colonization of erythromycin-susceptible and -Resistant Campylobacter jejuni. *Frontiers in Microbiology*.

[20] Pang A. S., Nathoo S., Wong S. L. (1991). Cloning and characterization of a pair of novel genes that regulate production of extracellular enzymes in Bacillus subtilis. *Journal of Bacteriology*.

[21] Toms A. V., Haas A. L., Park J.-H., Begley T. P., Ealick S. E. (2005). Structural characterization of the regulatory proteins TenA and TenI from Bacillus subtilis and identification of TenA as a thiaminase II. *Biochemistry*.

[22] Barison N., Cendron L., Trento A., Angelini A., Zanotti G. (2009). Structural and mutational analysis of TenA protein (HP1287) from the Helicobacter pylori thiamin salvage pathway – evidence of a different substrate specificity. *The FEBS Journal*.

[23] Begum A., Drebes J., Perbandt M., Wrenger C., Betzel C. (2011). Purification, crystallization and preliminary X-ray diffraction analysis of the thiaminase type II from Staphylococcus aureus. *Acta Crystallographica. Section F, Structural Biology and Crystallization Communications*.

[24] Toyama H., Nishibayashi E., Saeki M., Adachi O., Matsushita K. (2007). Factors required for the catalytic reaction of PqqC/D which produces pyrroloquinoline quinone. *Biochemical and Biophysical Research Communications*.

[25] Toyama H., Fukumoto H., Saeki M., Matsushita K., Adachi O., Lidstrom M. E. (2002). PqqC/D, which converts a biosynthetic intermediate to pyrroloquinoline quinone. *Biochemical and Biophysical Research Communications*.

[26] Hölscher T., Görisch H. (2006). Knockout and overexpression of pyrroloquinoline quinone biosynthetic genes in Gluconobacter oxydans 621H. *Journal of Bacteriology*.

[27] Haghjoo E., Galán J. E. (2007). Identification of a transcriptional regulator that controls intracellular gene expression inSalmonellaTyphi. *Molecular Microbiology*.

